The article "A Study on the Hedging Function of Gold in the Light of Economic Policy Uncertainty" was published in 2022. Journal: Comput Intell Neurosci.

# A Study on the Hedging Function of Gold in the Light of Economic Policy Uncertainty

**DOI:** 10.1155/2022/1556475

**Published:** 2022-06-16

**Authors:** Borui Xiao

**Affiliations:** Hainan University, Haikou, Hainan 570228, China

## Abstract

This paper focuses on the empirical analysis of the closing price of gold, the SSE Index, and the China Economic Policy Uncertainty Index by means of a GARCH model to study the main characteristics of their movements. The series of gold closing price returns are analysed for linkage using the current mainstream VAR model, so as to analyse and compare the hedging function of gold. The article selects the closing price of gold, the SSE Index, and the China News-Based EPU from June 2005 to June 2019 as the sample series for the study. The background of the study and the theoretical knowledge of VAR and GARCH models are first introduced, and then, the GARCH family model and statistical analysis methods are used to derive the respective movements of the log returns of gold closing price, SSE index log returns, and China News-Based EPU log volatilities. The results show that the movements of the closing price of gold, the SSE Index, and the China News-Based EPU have the characteristics of financial assets in general, such as spikes and thick tails, agglomeration, and leverage effects. For the empirical study of the linkage between the three, this paper first considers only three variables, namely gold closing price, SSE index, and EPU. In order to investigate whether there is a co-integration relationship between them, a vector autoregressive model is established, followed by the corresponding impulse response analysis and variance decomposition. The analysis of the linkage between the closing price of gold, the SSE index, and the EPU concluded that changes in the EPU had a greater impact on the changes in the closing price of gold, while changes in the SSE index had a smaller impact on the changes in the closing price of gold. Finally, the conclusion of this article is some advice to investors on gold investment.

## 1. Introduction

### 1.1. Background and Significance of the Study

Economic uncertainty is the inability of economic agents to predict if, when, and how the government will change existing economic policies. Gold is a special product with characteristics such as commodity, currency, and risk aversion. Risk aversion means that gold is a safe source of capital in times of major economic change and crisis. In the context of a worldwide economic recession, gold has become a “safe haven” for many investors. Due to the regular volatility of financial markets, investors worldwide are more than happy to add gold to their investment portfolios.

The risk-averse function of gold is usually applied in two situations.

Firstly, when global inflationary pressures increase, a rise in inflation means a reduction in the real value of paper money. Then, holding paper money will be at risk of devaluation and investors will invest relatively more in gold for the purpose of preserving its value.

Secondly, in the context of a shrinking world economy, the global economic downturn has also exacerbated the market fears caused by the global recession. As a result, investors prefer to protect themselves from risk by holding gold.

When the price of gold falls temporarily, discounts can be obtained until it rises again. If the price rises, there is the option of continuing to observe or analyse the need to sell gold based on the factors affecting the price of gold, which, although a long-term investment, are a viable way of maintaining the value of the asset.

Therefore, this paper builds on previous research and takes into account the current volatility in the capital markets to investigate the hedging and hedging of gold, with a view to compensating to some extent for the lack of research on risk-hedging assets in the capital markets.

### 1.2. Research Objectives

This paper will focus on the linkage between gold and Chinese economic policy uncertainty and examine the hedging function of gold. Empirical analysis will be conducted using VAR (vector of autoregression) and DARCH models. At the same time, the application of one model to the risk aversion capability of the gold market is an attempt and innovation of very practical importance to risk management in the gold market.

The following questions are addressed: (1) Is there a linkage between the gold price and the China Economic Policy Uncertainty Index? (2) Is there a correlation between the gold price and the SSE index? (3) Can gold be used as a hedging asset in extreme situations to bypass the sharp rise in economic policy uncertainty, and based on the above research, we analyse the hedging ability of gold and make more suitable investment recommendations to regulators and investors.

## 2. Review of the Literature

As an important component of commodities, gold's relationship with the economy and policy is at the heart of the debate. The relevant literature suggests that the disclosure of macroeconomic information has a significant impact on gold yields, with some studies, suggesting that the impact is more pronounced in times of economic contraction. Abken, for example, notes that the price of gold can change dramatically due to extreme political or economic uncertainty. [1] Ciner, Battenet al. suggest that gold became a refuge for the US stock market in the early 1990s and during the global financial crisis of 2008. [2]

Shafiee and Topal systematically collate and summarise the various factors that influence the price of gold and highlight that the short-term surge in gold prices is due to the fact that gold can act as a hedge against large fluctuations in traditional asset prices in times of financial market instability. [3] Batten et al. classify the real economy-related factors that may cause changes in commodity markets for precious metals such as gold, silver, platinum, and palladium into three types: variables that reflect the elasticity of the monetary environment, such as inflation rates and monetary aggregates; variables that reflect business prosperity, such as industrial GDP; and variables that reflect, for example, the exchange rate of the US dollar, returns on stock indices, and consumer confidence financial market variables such as the US dollar exchange rate, stock index returns, and consumer confidence indices. It was found that a certain degree of volatility in gold returns could be explained by the above economic variables. Chrtstie-David et al. investigated 23 macro indicators in the United States and found that the volatility of gold returns increased substantially over the reporting period, especially the volatility of gold returns in response to changes in capacity utilisation, CPI, and GDP. [4]

Cai et al. reported that the sale of the PBOC's gold reserves would lead to a fall in the price of gold. [5] Roache and Rossi's study of 11 macroeconomic indicators and 6 commodities including gold shows that nonagricultural wage indicators, consumer confidence indicators, and interest rates have a significant impact on gold, and that gold's reaction to bearish information reflects a value-protective, safe-haven nature and is therefore different from the other 5 commodities. [6] When gold is used as both a hedging asset and a safe-haven asset, Baur and Lucey present the first statistical test, showing that gold can be used as both a hedging and a safe-haven asset against the US dollar. [7] Elder et al. examined the relationship between gold returns, trading volume and volatility, and the publication of macro information and shows that gold has a significant and rapid response to economic information, with nonagricultural pay and nonconsumer orders being particularly influential in economic information. [8] In addition to this, gold is also sensitive to macro supply and demand information. Reboredo examines the correlation between daily data on the exchange rates of major international currencies against the US dollar and the gold price between 2000 and 2012. He extends Baur and Lucey's definition of safe-haven and hedging assets by arguing that safe-haven and hedging assets among financial assets can be measured by general and dynamic correlation coefficients. The results show that the gold price is generally correlated with the US dollar exchange rate, with a positive dynamic correlation coefficient, confirming Reboredo (2010) findings. [9].

In recent years, with the rapid development and expansion of capital markets, more and more scholars are studying how gold hedges risk and the information about it is becoming more comprehensive and complete. Xu verified that gold prices have a good hedging effect on the consumer price index as well as the US dollar index, and can be used as an indicator of inflation through Granger causality tests of the VEC model. [10] Yuan and Yang examined the feasibility of gold futures to hedge real foreign exchange risk. [11] Yang studied Shandong gold as a representative, and the results showed that: firstly, the SSE Composite Index is not the Granger cause of Shandong gold, while the international gold price is the Granger cause of Shandong gold; secondly, the impact effect of the international gold price on Shandong gold is extremely obvious, about twice that of the SSE Composite Index; thirdly, both the SSE Composite Index and the international gold price have a long-term impact on Shandong gold. Finally, the international gold price explains the rate of change in Shandong gold prices much more strongly than the SSE Composite Index. [12] Nian examined the effect of gold hedging in different countries from different perspectives in a comprehensive manner. The study shows that in the long run, gold investment has an anti-inflationary effect, and therefore, gold is an effective long-term hedge, especially during periods of accelerating inflation, when gold investment returns are particularly significant. [13] Hu and Zhao conducted an empirical analysis by building a GARCH-like model, revealing that there are heteroscedasticity effects, asymmetric spillover effects, and significant asymmetry in both the stock market and the gold market. [14] Ni and Yu used a BEKK-GARCH model to study the risk aversion ability of the Chinese gold market, and the results showed that gold only has certain hedging ability in the short term. [15]

In conclusion, gold is closely linked to the global real economy as well as to international financial markets. Gold is sensitive and responsive to timely macro information, suggesting that economic policy uncertainty has a significant impact on gold. We will judge whether gold can be used as a safe-haven asset to hedge against risks in the real economy or equity markets based on an examination of the linkage between gold and economic policy uncertainty.

## 3. Model Theory Research

This paper focuses on the hedging capacity of gold based on economic policy uncertainty. The relationship between the price of gold and future trading volume, and the policy uncertainty index is studied, and then, the covering capacity of gold is analysed based on the relationship between them. *Analysis of gold hedging capacity*. VAR models and GARCH-type models are used in this thesis, and this chapter provides a detailed introduction to VAR models and GARCH-type models.

### 3.1. VAR Model

#### 3.1.1. Definitions

If the n-dimensional time series {*Y*_*t*_},  *t* ∈ *T*,  *T*={1,2,…}, the *Y*_*t*_=*C*+*θ*_1_*Y*_*t*−1_+⋯+*θ*_*p*_*Y*_*t*−*p*_+*ε*_*t*_, satisfying, where *E*(*ε*_*t*_)=0, and *E*(*ε*_*t*_, *ε*_*t*_)={Ω*t*=*τ*/0*t* ≠ *τ*

This is then a *p*-order vector autoregressive mode.

If *ε*_*t*_ mutually independent and identically distributed and follows a normal distribution, then the stochastic process of the model is the autocorrelation process of the *P*-order vector, which is a standard VAR model, and the model is called VAR(P).

#### 3.1.2. Characteristics of the Standard VAR Model

1. Each component is an endogenous variable.
2. Each equation has the same explanatory variables.
3. *Y*_*t*_ the *p*-order lag of can then depict its dynamic structure that *Y*_*t*_. there is no response to variables prior to the *p* moment.
4. The VAR model is a simplified form of joint cubic equation.

#### 3.1.3. VAR Model Fixed Order

AIC (Akaike) and SC (Schwarz) guidelines are as follows:

(1) $$\begin{array}{c} \text{AIC}\left(p\right)=\text{Indet}\left(\hat{\sum p}\right)+\frac{2n^{2}p}{T},\\ \text{SIC}\left(p\right)=\text{Indet}\left(\hat{\sum p}\right)+\frac{n^{2}plnT}{T}. \end{array}$$

*N* is the vector size, *T* is the sample size, *p* is the lag order, det is the determinant of the solution matrix, and $\hat{\sum p}$ is an estimate of the residual vector covariance matrix for a lag length of *p*.

If the same lag order is chosen as for the univariate model, the following problems will arise.

1. The choice of criterion is subjective and arbitrary. Depending on the choice of criterion, the lag order may also vary.
2. The actual series can sometimes be a nonfinite dimensional process of random probability events, and although there are large quantities of time series that are not smooth, modelling the smooth time series with a finite lag length VAR model can lead to an exciting conclusion.
3. Even if the series is smooth, if the actual lag order is greater than *Q*, the correct lag length cannot be obtained.

### 3.2. Introduction to GARCH-like Models

GARCH-type models usually consist of two equations consisting of a conditional mean equation and a conditional variance equation. Before building a GARCH-type model, it is often necessary to test for the smoothness of the series and the ARCH effect. And the ARCH effect means that future fluctuations can be predicted using historical fluctuations. Therefore, GARCH-type models are often used to study time series volatility and correlation with historical data and to predict future data. Therefore, the conditional variance equation is extremely important, while the conditional mean equation is relatively straightforward. [16]

The mean value model is

(2) $$\begin{array}{c} r_{i}=\mu +\varepsilon_{i}, \end{array}$$

where *μ* is the unconditional mean, which is a constant, and *ε*_*i*_ is a random disturbance term. There are different criteria for classifying GARCH models: (1) according to the conditional mean equation, there are GARCH models and ARCH-mean models, that is, GARCH-M models; (2) whether they are symmetric, EGARCH, and RGARCH models

#### 3.2.1. Univariate GARCH

Bollerslev (1986) extended the scope of Engle's original model, the Arch model, by introducing a method in the Arch model that allowed the conditional variance to be transformed into an ARMA process.

The generalised ARCH or GARCH (*p*, *q*) is as follows:

(3) $$\begin{array}{c} h_{t}^{2}=\sum_{i=1}^{p}\beta_{i}\varepsilon_{t-i}^{2}+\sum_{i=1}^{q}\alpha_{i}h_{t-i}^{2}. \end{array}$$

The parameter *p* is also called the order of the ARCH term and the parameter *q* is the order of the GARCH term, *α*_0_ ≥ 0, *α*_1_ ≥ 0, *β*_*j*_ ≥ 0.

#### 3.2.2. GARCH-M Model

In addition to introducing the residual squared term of the conditional mean into the conditional variance equation, the conditional characteristics of the residual term can also be used as an explanatory variable affecting the {*Y*_*t*_} mean, and this type of model is called an ARCH mean model or GARCH-M model.

The GARCH-M model (Engle) and other academics proposed in 1988 to describe the change in risk premiums over time.

The GARCH-M model is as follows:

(4) $$\begin{array}{c} y_{t}=\beta +\delta h_{t}+\varepsilon_{t},\\ h_{t}^{2}=r+\alpha \sum_{j=1}^{i}\varepsilon_{t-j}^{2}+\sum_{j=1}^{i}h_{t-j}^{2}. \end{array}$$

#### 3.2.3. Exponential GARCH: E-GARCH

The E-GARCH (exponential GARCH) model proposed by Nelson (1991) is as follows:

(5) $$\begin{array}{c} \ln\;h_{t}^{2}=\alpha_{0}+\sum_{i=1}^{p}\alpha_{i}\frac{\left|\varepsilon_{t}-1\right|}{h_{t}-1}+\sum_{i=1}^{q}\beta \;\ln\;h_{t-i}^{2}+\sum_{k=1}^{r}\lambda_{k}\frac{\varepsilon_{t-k}}{\sqrt{h_{t-i}}}. \end{array}$$

*λ* < 0, then the existence of a leverage effect is indicated. *λ* ≠ 0, impact of the shock is the asymmetric.

#### 3.2.4. The TGAECH Model

*Simple modified symmetry*. The GAECH framework can describe the consequences of asymmetries of positive and negative disturbances. The TGAECH model proposed by Zakoian (1990) and Glosten, Jaganathan, and Runkle (1993) is as follows:

(6) $$\begin{array}{c} h_{t}^{2}=\alpha_{0}+\sum_{i=1}^{p}\rho_{i}h_{t-i}+\sum_{i=1}^{q}\alpha_{i}\varepsilon_{t-i}^{2}+\gamma \varepsilon_{t-1}^{2}d_{t-1}. \end{array}$$

## 4. Data Selection, Description, and Changes

### 4.1. EPU and Data Selection

The Economic Policy Uncertainty Index, or EPU Index for short, is an index of economic policy uncertainty. It is compiled by Scott R. Baker, Nicholas Bloom, and Steven J. Davis and is generally used to reflect economic and policy uncertainty in the world's major economies. Their research has shown that the EPU Index has an apparently contradictory relationship with actual measures of macroeconomic indicators and can even explain to some extent the dramatic fluctuations in equity markets. In China, the EPU Index has a positive relationship with the bond market and a negative relationship with the stock market.

In this paper, gold (Au *T* + *d*) closing price, volume, turnover, weighted average price, position, SSE Index (SSEC), and Economic Policy Uncertainty Index (China News-Based EPU) are selected as the research samples. The frequency of the data selected is monthly, spanning 14 years from June 2005 to June 2019, with 169 sets of observations from the CSMAR database. Since the closing price, volume, turnover, weighted average price, and position of gold (Au *T* + *d*) are identical to the modelling process of the SSE Index and the Economic Policy Uncertainty Index, this paper will only model the closing price return rt with the SSE Index volatility *r*_*s*_ and the Economic Policy Uncertainty Index volatility *r*_*e*._

As shown in Figure 1, the overall trend in the volatility of the closing price of gold has been up and then down, rising from June 2005, peaking in November 2011, and then gradually declining.

The data were all logarithmically processed to obtain a series of log returns (log volatilities).

(7) $$\begin{array}{c} \text{Return}=\ln\left(p_{t}\right)-\ln\left(p_{t-1}\right). \end{array}$$

### 4.2. An Empirical Study of the Volatility Characteristics of Gold Closing Prices

There are many modelling approaches to empirically analyse the characteristics of changes in financial assets, and here, we have chosen the GARCH family of models. In this chapter, the GARCH (1, 1), GARCH-M, EGARCH, and TGARCH models are used to analyse the patterns of change. The model coefficients are estimated using great likelihood, and correlations are tested using the ARCH-LM method. The selection of optimality for each model is judged using the AIC and SC criteria.

#### 4.2.1. Basic Processing of Gold Closing Price Data

*(1) Descriptive Statistics of Gold Closing Prices*. 

Table 1 shows that the skewness is −0.352225, so the log return series of gold closing prices is left skewed (the skewness of the normal distribution is 0); the kurtosis is 4.010878 and 4.010878 > 3, and 3 is the kurtosis of the normal distribution, so we can conclude that the log return series of gold closing prices has “sharp peaks and thick tails.” Jarque–Bera is a *χ*^2^ statistic that is often used to test whether a series follows a normal distribution. At the same time, the statistical properties of the log returns indicate that the original hypopaper is rejected and the distribution is not normal.

This paper therefore establishes a GARCH model, which is able to balance the time-varying characteristics that the sample data have. Based on the findings, it can be seen that the gold yield series does not exactly obey the standard normal distribution. In this case, based on the results of previous scholars, using a distribution can better fit the distribution characteristics of the sample data. So, as to arrive at optimal empirical results, this paper also examines the sample data using the GARCH equation under a *T* distribution. Ultimately, however, one must also take into account that the *T* distribution of the sample series is more consistent with the normal distribution, and this paper then proceeds to simulate a model based on the normal distribution. Based on the fact that after the normality test has been done above, the statistical characteristics of the time series that need to be examined if a GARCH model is to be built, this paper will therefore do a smoothness test, a data autocorrelation test, and an effects test on the sample time series.

*(2) Statistical Characteristics of Gold Closing Prices and Correlation Tests*. The statistical analysis above shows that the log return series of the closing price of gold has the characteristics of a spike with a thick tail and its volatility series does not obey a normal distribution as known by the chemical statistics. To fully illustrate its disobedience to a normal distribution, a normal QQ plot is plotted, see Figure 2.

As shown in Figure 2, a large number of points are scattered outside the straight line of the normal distribution; thus, the actual distribution of the log return series of gold closing prices has a thick tail. The ADF unit root test for its smoothness, without the intercept term and without the time trend term, is shown in Figure 3, and the *P*-value of the ADF test for the log return time series of gold closing prices is 0, rejecting the null hypopaper of containing a unit root, which indicates that the series is stable.

*(3) Autocorrelation Test*. It is a test for serial autocorrelation. Many distributions of returns are not only kurtic and skewed and move over time, but the returns of successive adjacent periods are not necessarily independent of each other, a phenomenon known as autocorrelation of a return series. Sequences are autocorrelated because of the inertia and stickiness of their own series, which leads to correlation between residuals. Therefore, in order to better create a VAR-GARCH model, this paper needs to examine the autocorrelation of the return series.

The yield series were tested with the autocorrelation function (ACF) and the partial correlation function (PACF), as shown in Figure 4, after which the results of the study were obtained for the lags to maturity: rt has 6th-order autocorrelation.

Based on the previous analysis, it is clear that the log return series of the closing price of gold is smooth, with clustering of its fluctuations and possible conditional heteroscedasticity, a distinctive feature of the GARCH model is that it allows the time series to have time-varying conditional variance.

*(4) Conditional Heteroscedasticity Test and ARCH Test*. Assuming that the residuals of the log return series of the closing price of gold obey a normal distribution (Bollerslev and Wooldridge have done a study where, as long as the mean coincident variance equation is set in the correct form, the maximum-likelihood estimates are still consistent even if the assumption of conditional normal distribution does not hold), a maximum-likelihood estimate of the log return series of the closing price of gold with a 6th-order lag is performed, and then, ARCH effect test was then performed on its residual term. The results are shown in Figure 5. The *P*-value of the LM statistic is 0.0048, which is smaller than the significance level of 0.05. This means that the log return series of the closing price of gold contains a higher order ARCH effect and can be modelled using a GARCH model.

#### 4.2.2. GARCH-like Model Analysis

1. The GARCH (1, 1) model, the GARCH-M model, the EGARCH model, and the TGARCH model are modelled assuming a t-distribution of the error term of the log return on the closing price of gold.

GARCH (1, 1) model with mean equation is as follows:

(8) $$\begin{array}{c} RT_{t}=0.002354+0.192813RT_{t-6}+{\hat{u}}_{t}\left(0.779734\right)\left(2.492220\right),\\ R^{2}=0.33933,\\ DW=2.176027. \end{array}$$

Corresponding GARCH (1,1) equation is as follows:

(9) $$\begin{array}{c} \sigma_{t}^{2}=0.0000503+0.274179u_{t-1}^{2}+0.708382\sigma_{t-1}^{2}\left(0.973159\right)\left(2.347141\right)\left(9.371286\right). \end{array}$$

GARCH-M model with mean equation is as follows:

(10) $$\begin{array}{c} RT_{t}=-0.353251+0.157942RT_{t-6}+7.543124\sqrt[{2}]{\sigma_{t}^{2}}+{\hat{u}}_{t}\\ \left(-0.817324\right)\left(2.173317\right)\left(0.809165\right)\\ R^{2}=0.056204\;DW=2.086611. \end{array}$$

GARCH-M equation is as follows:

(11) $$\begin{array}{c} \sigma_{t}^{2}=0.001544+0.025769u_{t-1}^{2}+0.294520\sigma_{t-1}^{2}\left(1\text{.}72235\right)\left(\text{0.}751752\right)\left(\text{0.}856811\right). \end{array}$$

EGARCH model with mean equation is as follows:

(12) $$\begin{array}{c} RT_{t}=0.002639+0.200228RT_{t-6}+{\hat{u}}_{t}\left(\text{0.}812466\right)\left(2\text{.}547833\right)\\ R^{2}=0.034358\;DW=2.19355. \end{array}$$

EGARCH equation is as follows:

(13) $$\begin{array}{c} \ln\left(\sigma_{t}^{2}\right)=-0.941444+0.497627\left|u_{t-1}/\sigma_{t-1}\right|-0.000486u_{t-1}/\sigma_{t-1}+0.910791\;\ln\left(\sigma_{t-1}^{2}\right)\\ \left(2.180059\right)\left(2.835271\right)\left(0.005617\right)\left(15.33532\right). \end{array}$$

TGARCH model with mean equation is as follows:

(14) $$\begin{array}{c} RT_{t}=0.002212+0.192738RT_{t-6}+{\hat{u}}_{t}\left(\text{0.}714730\right)\left(\text{0.}0077217\right),\\ R^{2}=0.033669\;DW=2.171473. \end{array}$$

TGARCH equation is as follows:

(15) $$\begin{array}{c} \sigma_{t}^{2}=0.0005+0.263328u_{t-1}^{2}+0.025729u_{t-1}^{2}d_{t-1}+0.747799\sigma_{t-1}^{2}\\ \left(0.966826\right)\left(1.976846\right)\left(0.155165\right)\left(9.28640\right). \end{array}$$

The specific GARCH estimation model was determined by selecting the GARCH model that corresponds to when the AIC and SC values are minimised according to the Akaike information criterion and the Schwarz criterion, that is, the AIC criterion and the SC criterion. Using the graphs above, Table 2 can be obtained.

In summary, by comparing the GARCH (1,1) model, GARCH-M model, EGARCH model, and TGARCH model for fitting parameters, according to the Akaike information criterion and Schwarz criterion, that is, AIC criterion and SC criterion, the GARCH (1,1) model, AIC value, and SC value reach the minimum, and GARCH (1,1) for the three sets of data GARCH (1,1) was chosen as the best fit for the residual series of log returns.

GARCH (1, 1) model with mean equation is as follows:

(16) $$\begin{array}{c} RT_{t}=0.002354+0.192813RT_{t-6}+{\hat{u}}_{t}\left(0.779734\right)\left(2.492220\right),\\ R^{2}=0.33933,\\ DW=2.176027. \end{array}$$

Corresponding GARCH (1,1) equation is as follows.

(17) $$\begin{array}{c} \sigma_{t}^{2}=0.0000503+0.274179u_{t-1}^{2}+0.708382\sigma_{t-1}^{2}\left(0.973159\right)\left(2.347141\right)\left(9.371286\right). \end{array}$$

The coefficients of both the ARCH and GARCH terms in the GARCH (1,1) equation are significant, and the sum of the coefficients of the ARCH and GARCH terms are 0.274179 + 0.708382 = 0.982561 < 1, satisfying the constraints on the parameters. Since the sum of the coefficients is very close to 1, it means that this conditional variance is subject to continuous shocks; that is, it has great predictive power for the future.

### 4.3. An Empirical Study of the Volatility Characteristics of the SSE Index

Similar to the empirical study of the volatility characteristics of the closing price of gold in 4.2 above:

#### 4.3.1. Descriptive Statistics and Trends of the SSE Index

From Table 3, we can find that the skewness is −0.64021, so the series is left-skewed (the skewness of the normal distribution is 0); the kurtosis is 4.801406 > 3, thus determining that the SSE log return series is characterised by “sharp peaks and thick tails.” The Jarque–Bera statistic also shows the rejection of the normal distribution hypothesis.  Figure 6 shows the trend of the log returns of the SSE index.

#### 4.3.2. Statistical Characteristics of the SSE Index and Correlation Tests

The ADF unit root test for its smoothness, without the intercept term and without the time trend term, can be seen in Figure 7, where the ADF test *P*-value for the log return time series of the SSE index is 0, rejecting the null hypopaper of containing a unit root, then indicating that the series is smooth.

#### 4.3.3. Autocorrelation Test

The SSE log return series was tested for autocorrelation function (ACF) and partial correlation function (PACF), as shown in Figure 8, after which the findings for the lags to maturity were obtained: rs has 4th-order autocorrelation.

#### 4.3.4. Conditional Heteroscedasticity Test and ARCH Test

As can be seen from Figure 9, the LM statistic *P*-value of 0.9316 is significantly greater than the significance level of 0.05, which would indicate that there is no higher order ARCH effect in the effective exchange rate log return series and that the GARCH model cannot be used further to study its movement. This can be attributed to the data selection problem; the GARCH family of models is generally applicable to high-frequency data, and only monthly data from June 2005 to June 2019 were chosen for this study, and the sample size is far less than high-frequency data, so the model simulation effect may not be ideal. But it does not negate the fact that SSE index movements are agglomerative and leveraged. From the statistical description of SSE index fluctuations in the previous section and the series trend graph, the trend of SSE index movements can still be derived.

### 4.4. Empirical Study of EPU Volatility Characteristics

Similar to the empirical study of the volatility characteristics of the closing price of gold in 4.2 above:

#### 4.4.1. Descriptive Statistics and Trends in EPU

From Table 4, we can see that the skewness is −0.15141, so the EPU rate of change return series is left-skewed (the skewness of the normal distribution is 0); the kurtosis is 4.135106 > 3, respectively, which leads to the conclusion that the EPU rate of change series is characterized by “sharp peaks and thick tails.” The Jarque–Bera statistic also shows that the assumption of a normal distribution is rejected.  Figure 10 shows the trend of the EPU rate of change.

#### 4.4.2. Statistical Characteristics of EPU and Correlation Test

When the ADF unit root test for its smoothness is performed, without the intercept term and without the time trend term, it can be seen from Figure 11 that the *P*-value of the ADF test for the log return time series of the SSE index is 0, which rejects the null hypopaper of containing a unit root, and then indicates that the series is smooth.

#### 4.4.3. Autocorrelation Test

Autocorrelation functions (ACF) and partial correlation functions (PACF) were performed on the EPU rate of change series, as shown in Figure 12, after which findings were obtained for the lags due to re with 1st- and 2nd-order autocorrelation.

#### 4.4.4. Conditional Heteroscedasticity Test and ARCH Test

As can be seen from Figure 13, the LM statistic *P*-value of 0.3436 is significantly greater than the significance level of 0.05, which would indicate that there is no higher order ARCH effect in the effective exchange rate log return series and that the GARCH model cannot be used further to study its movement. This can be attributed to the data selection problem; the GARCH family of models is generally applicable to high-frequency data, and only monthly data from June 2005 to June 2019 were chosen for this study, and the sample size is far less than high-frequency data, so the model simulation effect may not be ideal. However, it does not negate the fact that the SSE index movements have a clustering and futile pole effect. From the statistical description of SSE index fluctuations in the previous section and the series trend graph, the trend of SSE index movements can still be derived.

## 5. Empirical Analysis of the Linkage between the Closing Price of Gold and the SSE Index and the China Policy Uncertainty Index

As China's economic system continues to reform and the gold market process advances, many changes have occurred in China's economic environment, which inevitably lays the foundation for further strengthening the linkage between the closing price of gold and the SSE and the China Policy Uncertainty Indices. Chapter 3 describes some common GARCH models, and in Chapter 4, we empirically analyse the movements of the log returns of the gold closing price, the log returns of the SSE, and the log volatility of the China Policy Uncertainty Index, thus providing a clearer picture of their patterns of movement. This chapter builds on the previous chapters on the linkages between the closing price of gold and the SSE and China Policy Uncertainty Index linkages. The first step is to test whether there is a long-run co-integration relationship between the gold closing price and the SSE and China Policy Uncertainty Indices, establish a vector autoregressive (VAR) model, and conduct impulse response analysis. The Johansen test is used to establish the co-integration equation and vector error correction model for the long-term equilibrium relationship between the closing price of gold and the China Policy Uncertainty Index; the impulse response and variance decomposition are used to analyse the direction and extent of their influence.

As can be seen from Chapter 4, both sets of data, the log return on the closing price of gold, the log return on the SSE, and the rate of change of the EPU are non-normally distributed series.

### 5.1. ADF Test

In order to avoid pseudoregression, we need to first perform a unit root test on the data to determine the stability of the data. The results of the ADF test are shown in Table 5, where c, t, and k represent the constant term, the time trend term, and the optimal lag order of the ADF test, respectively, and the *P*-value is obtained from the AIC minimum principle.

As can be seen from Table 5, rt, rs, and re are all smooth series at the 5% level of significance and no co-integration test is required.

### 5.2. Determination of the Lag Order

As the lag order affects the stability of the model, it is important that the lag order is set correctly before modelling. The longer the lag order, the better the fit of the model, but higher lag orders also entail a higher loss of degrees of freedom. Here, we will first determine the optimum number of lags. There are various criteria for judging the lag order, such as likelihood ratio (LR), AIC, and SC. The results of the tests are shown in Figure 14.

From Figure 14, it can be seen that the best lag order is 2; that is, the optimal lag order is set to 2.

### 5.3. Granger Causality Test

A further Granger causality test was done on the trivariate series of the gold closing price and the SSE and China Policy Uncertainty Indices. As shown in Figure 15, the probability that rs is not rt's Granger causality is 0.6671, which cannot reject the original hypopaper at the 5% significant level; that is, rs has no predictive power for rt; the probability that re is not rt's Granger causality is 0.0400, which rejects the original hypopaper at the 5% significant level; that is, re has predictive power for rt.

### 5.4. VAR Model Development and Analysis of Results

A VAR (2) model is developed, and its estimation results (Table 6) are as follows:

(18) $$\begin{array}{c} RT=-0.0794677159514*RT\left(-1\right)-0.0127198550478*RT\left(-2\right)-0.0.386137808512*RS\left(-1\right)\\ +0.0189136417895*RS\left(-2\right)+0.00829161885013*\left(-1\right)-0.0154847640009*\\ RE\left(-2\right)+0.00677555375429. \end{array}$$

The *F*-test values from the VAR(2) equation are coincidentally 83.24589711, respectively, which shows that the equation is estimated to be significant. From the *T*-statistic of each coefficient of the equation, the absolute value of the coefficient of re(−2) is larger and more significant than the T-statistic of 1.64 at the 10% level, while the coefficients of the remaining variables are not significant, indicating that the log return of the closing price of gold is mainly influenced by the 2nd-order lag of EPU. However, when analysed by the magnitude of the coefficients, a 1% change in the 2nd-order lag of EPU results in a 1.549% change in the log return of the closing price of gold. This shows that there is a linkage between the log return on the closing price of gold and the rate of change of the EPU.

### 5.5. Impulse Response Analysis

#### 5.5.1. Model Stability Tests

Before impulse response analysis, the stability of the established VAR (2) model needs to be tested. The impulse response analysis will only be more meaningful if the model is stable. This section uses the eigenroot test (AR) method, which means that the model is stable if the reciprocal of all the root modes of the VAR model is less than 1; that is, the eigenroots of the model all lie within the unit circle. The results are shown in Figure 16, where all the characteristic roots of the model lie within the unit circle, which indicates that the model is stable and allows for impulse response analysis.

#### 5.5.2. Response Analysis

The impulse response function analysis method is used to describe the response of an endogenous variable to a shock caused by an error term; that is, the effect on the current and future values after a shock of a standard deviation size is applied to the random error term. As can be seen from Figure 17, rt's shock to itself slowly becomes smaller from period 1, reaches a minimum in period 2, is an assignment, then slowly becomes larger, crosses 0, reaches an extreme value in period 8, and converges to 0 thereafter; rs's shock to rt starts at 0 in period 1, gradually becomes smaller, reaches a minimum in period 2, and gradually becomes larger across 0, reaches a maximum in period 3, and then fluctuates up and down of convergence with 0; re's shock to rt, starts at 0 in the first period, gradually becomes larger, reaches a maximum in the second period, and gradually becomes smaller across 0, reaches a minimum in the third period, and then fluctuates up and down convergence with 0.

### 5.6. Variance Decomposition

The basic idea of variance decomposition is to decompose the fluctuations of all the variables in the system (*k*) into *k* components associated with each equation's new interest by their causes, thus obtaining the relative importance of the new interest to the model's endogenous variables.

As can be seen from Table 7 and Figure 18, in period 1, a perturbation of rt acts entirely on rt itself, but gradually decreases over time, but more slowly, and by period 10, the contribution is still 95.24788. In the process of rt being gradually weakened by its own perturbation, the contribution of rs and re to the effect of rt gradually increases, with re increasing more, and in period 10, it increases to 4.75212. However, relative to the 95.24788 contribution of rt to itself, the impact of rs and re on rt is small; that is, its transmission mechanism is hindered.

Therefore, the variance decomposition of the log return of the closing price of gold with the log return of the SSE Index and the rate of change of the EPU shows that although there is a linkage between them, the linkage is not strong. The impact of the change of the EPU on the change of the closing price of gold is stronger, and the impact of the change of the SSE Index on the change of the closing price of gold is weaker.

## 6. Conclusions and Recommendations

The article begins with a detailed description of the models used and then applies these models to an empirical analysis of gold closing price movements, focusing on the linkages between gold closing prices and the SSE Index and the China Economic Policy Uncertainty Index. The general idea of the empirical analysis section is as follows: (1) to carry out an empirical analysis of the closing price of gold, the SSE Index, and the China Economic Policy Uncertainty Index, and to study the main characteristics of their movements; (2) to analyse the linkage between the closing price of gold and the SSE Index and the China Economic Policy Uncertainty Index. The above study leads to the empirical results. The autoregressive model shows that there is a linkage relationship between the China Economic Policy Uncertainty Index and the closing price of gold. Impulse response analysis was carried out, and the direction of change between them was derived from the impulse response results. Given a standard deviation shock to the SSE Index, the direction of change of the gold closing price was negative and then positive and finally stabilised, and given a standard deviation shock to the China Policy Uncertainty Index, the direction of change of the gold closing price was positive, first increasing then decreasing until it stabilised. The impact of the SSE on the closing price of gold is greater than the impact on the China Policy Uncertainty Index. From the variance decomposition, it is obvious that the closing price of gold explains itself to the greatest extent, the SSE index, and China economic policy uncertainty index explain the closing price of gold to a lesser extent, while the China economic policy uncertainty index explains the closing price of gold to a greater extent.

The hedging of gold should be adjusted accordingly to the economic policy environment in order to ultimately preserve and hedge risk. The increased demand for the protective properties of gold is also a result of the dynamics of the gold market, which developed after the dematerialisation of gold as it met the demand for protected investments, which was changed by investors' distrust of credit currencies. Gold is one of the most liquid of all asset classes around the world and is the only asset that does not need to be liquidated through domestic credit or corporate debt. People readily accept gold, which tends to move faster than other assets, for large transactions. Not only can gold be sold on the financial markets, but also it is increasingly becoming a recognised collateral, thus further increasing its liquidity and protection function.

## Figures and Tables

**Figure 1:** Gold closing price, SSE, and EPU chart, June 2005–June 2019.

**Figure 2:** Normal QQ plot of the log return series for the closing price of gold.

**Figure 3:** Smoothing test for the log return series of the closing price of gold.

**Figure 4:** Autocorrelation test for log return series of gold closing prices.

**Figure 5:** ARCH-LM test table for the log return series of the closing price of gold.

**Figure 6:** Trend in log returns of the SSE Index.

**Figure 7:** ADF test for the log return series of the SSE Index.

**Figure 8:** Log return series autocorrelation test for the SSE Index.

**Figure 9:** ARCH-LM test table for the log return series of the SSE index.

**Figure 10:** Trends in the rate of change of EPU.

**Figure 11:** ADF test for EPU's log-volatility series.

**Figure 12:** Log volatility series autocorrelation test for EPU.

**Figure 13:** ARCH-LM test table for log volatility series of EPU.

**Figure 14:** Optimal lag order test.

**Figure 15:** Granger causality test results.

**Figure 16:** VAR (1) unit root test.

**Figure 17:** Impulse response diagram.

**Figure 18:** Variance decomposition plot for rt.

**Table 1:** Descriptive statistics for log returns on the closing price of gold.

	Average value	Maximum value	Minimum value	Standard deviation	Skewness	Kurtosis	Jarque–Bera statistic
Rt	0.006159	0.122465	−0.172233	0.047912	−0.352225	4.010878	10.69012

**Table 2:** GARCH model information criterion test results.

	GARCH(1,1) model	GARCH-M model	EGARCH model	TGARCH model
AIC	−3.253605	−3.332335	−3.342026	−3.320252
SC	−3.120745	−3.218454	−3.209165	−3.187391

**Table 3:** Descriptive statistics of log returns of SSE indices.

	Average value	Maximum value	Minimum value	Standard deviation	Skewness	Kurtosis	Jarque–Bera statistic
Rs	0.00611	0.242526	−0.28278	0.082856	−0.64021	4.801406	34.39535

**Table 4:** Descriptive statistics for the rate of change of EPU.

	Average value	Maximum value	Minimum value	Standard deviation	Skewness	Kurtosis	Jarque–Bera statistic
Re	0.13074	1.656059	−1.76689	0.480191	−0.15141	4.135166	9.719588

**Table 5:** ADF test results.

Variables	ADF values	Test form (*c*,*t*,*k*)	*P*-value	Stability
rt	−13.9385	(0, 0, 0)	0.001	Stable
rs	−11.3134	(0, 0, 0)	0.001	Stable
re	−17.4042	(0, 0, 1)	0.001	Stable

**Table 6:** Coefficients and t-statistics of the VAR model.

	RT(−1)	RT(−2)	RS(−1)	RS(−2)	RE(−1)	RE(−2)	*C*
Coefficient	−0.070468	−0.01272	−0.03861	0.018914	0.008292	−0.01549	0.006776
	0.08046	0.07889	0.04595	0.04583	0.00836	0.00836	0.00375
*T*-statistic	[−0.87583]	[−0.16124]	[−0.84036]	[0.41265]	[0.99159]	[−1.85214]	[1.80610]

**Table 7:** Variance decomposition table.

Period	S.E.	RT	RS	RE
1	0.047576	100.0000	0.000000	0.000000
2	0.047978	98.90152	0.648567	0.449911
3	0.048668	96.13051	0.897432	2.972055
4	0.048752	95.81839	0.899005	3.282602
5	0.048820	95.57686	0.902164	3.520980
6	0.048883	95.32839	0.899865	3.771741
7	0.048885	95.32503	0.903522	3.771446
8	0.048901	95.26552	0.903542	3.830940
9	0.048904	95.25221	0.903639	3.844147
10	0.048906	95.24788	0.903966	3.848156
Cholesky ordering	: RT RS RE			

## Data Availability

The data are available from the corresponding author upon request.
